The article "Quality of Life and PTSD Symptoms, and Temperament and Coping With Stress" was retracted in 2020. Reason: duplicate publication.

# Quality of Life and PTSD Symptoms, and Temperament and Coping With Stress

**DOI:** 10.3389/fpsyg.2018.02072

**Published:** 2018-11-01

**Authors:** Agnieszka Burnos, Kamilla M. Bargiel-Matusiewicz

**Affiliations:** Faculty of Psychology, University of Warsaw, Warsaw, Poland

**Keywords:** malignant neoplasm, cancer, quality of life, temperamental traits, stress coping styles, PTSD

## Abstract

Due to advances in medicine, a malignant neoplasm is a chronic disease that can be treated for a lot of patients for many years. It may lead to profound changes in everyday life and may induce fear of life. The ability to adjust to a new situation may depend on temperamental traits and stress coping strategies. The research presented in this paper explores the relationships between quality of life, PTSD symptoms, temperamental traits, and stress coping in a sample of patients diagnosed with cancer. One hundred and twenty nine participants aged 24–81 years, 69 females diagnosed with breast cancer and 60 males diagnosed with lung cancer completed Formal Characteristics of Behavior – Temperament Inventory, Coping Inventory for Stressful Situations, PTSD Inventory, and Quality of life SF-36 questionnaire. Higher level of emotional reactivity and higher level of perseveration was associated with lower emotional quality of life. Higher level of emotion oriented-coping and higher level of avoidant-distracted coping was associated with higher level of PTSD symptoms. Emotion-oriented coping and avoidant-distracted coping are ineffective in dealing with stress in the case of patients diagnosed with cancer, because they are associated with a higher level of PTSD symptoms. The significance of temperamental traits for quality of life in the situation of the patients is marginal. Control of specific factors concerned with current health and treatment status is needed the future research.

## Introduction

Malignant neoplasm is still one of the leading causes of mortality, but advances in medicine made it possible to treat it or to prolong life of people diagnosed with cancer (Heymach et al., 2018). For many people, it is a chronic disease that can be treated for many years and as such it leads to new issues such as stress related to one’s health condition and possible failure of treatment, the necessity to adjust to the illness, emotional, cognitive, and psychological effects of the disease and treatment and changes in family system and social environment of chronically ill people (Rzeszutek et al., 2015; Ahmad et al., 2017).

Based on the definition of World Health Organization (1995) quality of life includes one’s evaluation of physical health, emotional state, independence, and relations with social environment. Better quality of life reflects adaptation to the new situation of living with demands and restrictions resulting from health condition and treatment. It is also an evidence of adaptive psychological dealing with the consequence of illness in the form of a reduced range of many abilities. A chronic disease changes the way of functioning in many areas and the ability to adjust to a new situation may depend on many factors. Temperamental traits and stress coping strategies may be some of them (Husson et al., 2017). Temperamental traits may act as moderators of life events’ impact increasing or decreasing their stimulating value (Strelau, 2006). They may also affect coping strategies applied to stressful situations.

Patients diagnosed with malignant neoplasm have to deal with various sources of stress, the illness itself, much limited control over the illness, feel of guilt (especially if they have smoked cigarettes), depression, mood swings, fear of dying, sleep disorders, undergoing surgery, uncertain prognosis, side-effects of chemotherapy, changes in personal, family, and professional life. The treatment is usually long-term and painful, and it leads to a remission and not to a complete recovery. The side-effects may be difficult to bear. Sometimes loss of limbs and disability are possible. There are cases when separation with family is inevitable. Life opportunities are limited for shorter or longer periods of time. There is also risk of stigmatization (Lehto, 2017). Many patients report chronic distress or delayed distress especially during the first 12 months following the diagnosis (Gil et al., 2012; Myers et al., 2013; Zebrack et al., 2014). Their quality of life is lower than in the general population (Derogatis et al., 1983) while the prevalence of psychiatric disorders is higher (Gopalan, 2013).

The way of coping with stress affects quality of life more than the stress itself (Ogińska-Bulik and Juczyński, 2010). People differ in their coping strategies applying more task-oriented, emotion-oriented, or avoidant approach (Endler and Parker, 1990). Coping styles that may be considered ineffective in usual functioning may be beneficial in specific conditions.

Patients diagnosed with cancer feel better when they receive adequate social support (Karademas et al., 2007; Deb and Deka, 2015; Haugland et al., 2016). Coping approach coping was found to be positively related to positive health behavior changes and avoidant coping to negative behavior changes (Park et al., 2008). On the other hand, it was also found that avoidant repressive coping may actually be beneficial in terms of immunity to acute stress disorder in cancer patients (Pedersen and Zachariae, 2010), but this area needs more research. Avoidant coping strategies were found to be associated with poorer well-being, however, the severity of cancer was found to be a moderator of this relationship (Costanzo et al., 2006). Temperamental traits and coping strategies were also analyzed as predictors of PTSD symptoms and quality of life in the sample of patients after myocardial infarction (Burnos, 2018, unpublished).

Malignant neoplasm is potentially a life-threatening illness. In consequence, receiving the diagnosis of cancer is a very stressful event (Sellick and Edwardson, 2007). Patients usually think stereotypically that their prognosis is poor and even successful treatment does not prevent recurrence of the disease (Sheridan and Radmacher, 1992). The experience may be considered as a traumatic event and afterwards may result in PTSD symptoms (Arnaboldi et al., 2014; Moye and Rouse, 2015). Perceived life threat, serious medical diagnoses and following treatment were found to be factors that induced both PTSD symptoms and increased distress (Tedstone and Tarrier, 2003). It was more strongly related to psychological distress than to the actual cancer stage (Laubmeier and Zakowski, 2004). In many studies, conducted among others on victims of disasters and catastrophes it came out that traits such as emotional reactivity, perseveration, and activity are significant moderators of psychological consequences (e.g., PTSD) of experienced trauma (Strelau, 2008). Research also suggest that low-emotional reactivity may act as a specific protector against cancer trauma symptoms in adults (Oniszczenko and Laskowska, 2014). There is also possibility for post-traumatic growth. Cancer-specific stress was found to be positively correlated with PTG (Groarke et al., 2017; Occhipinti et al., 2015).

The complexity of the issue demands leaving the unidimensional medical model and conducting research based on biopsychosocial model which emphasizes physical, psychological, and social integrity of a human being. The process of recovery or dealing with progressive disease depends on many factors. Effective pharmacotherapy or successful surgery is crucial, but psychological and social processes are also very important.

### Current Study

This paper combines four different components of dealing with cancer such as the trauma of being diagnosed with life threatening-illness and being subject to aggressive treatment inducing intensive side-effects. The components are as follows: temperament, coping styles, PTSD symptoms, and quality of life. Temperament and coping styles are assumed to be predictors of PTSD symptoms and quality of life. According to this model temperamental traits and more or less adaptable, stress coping can result in PTSD symptoms or with adequate dealing with the trauma. Quality of life changes accordingly to one’s ability to deal with the new situation.

The research presented in this paper tries to explore the relationship between quality of life and level of PTSD symptoms of people diagnosed with cancer and psychological factors such as temperamental traits and stress coping. The results are than compared to the data obtained from the sample of patients after myocardial infarction.

There were four hypotheses formulated:

H1. There is relationship between temperamental traits and PTSD symptoms.
H2. There is relationship between stress coping and PTSD symptoms.
H3. There is relationship between temperamental traits and quality of life.
H4. There is relationship between stress coping and quality of life.

## Materials and Methods

### Participants

One hundred and twenty nine participants who were diagnosed with malignant neoplasms were recruited for the study. Women participating in the study were diagnosed with breast cancer. Men were diagnosed with lung cancer. These two were chosen because, according to National Cancer Registry in Poland, breast cancer is the most frequent malignancy in the population of women, while lung cancer is the most frequent malignancy in the population of men. Patients in terminal stage under palliative care were not included in the sample. Participation took place when they were hospitalized. It was voluntary and anonymous. The participants were not remunerated. Informed consent was obtained from all individual participants included in the study.

The research project was accepted by the local Research Ethics Committee at the Faculty of Psychology, University of Warsaw.

### Assessment

Temperament traits were assessed with the Formal Characteristics of Behavior – Temperament Inventory, FCB-TI (Strelau and Zawadzki, 1995). This questionnaire measures six temperament traits: briskness, perseveration, sensory sensitivity, emotional reactivity, endurance, and activity and is based on Regulative Theory of Temperament (RTT) of Strelau (1996), which concentrates on formal aspects of behavior comprising energetic and temporal characteristics composed of such traits as: sensory sensitivity, emotional reactivity, endurance, and activity (energetic aspect), briskness, and perseveration (temporal combustion). Sensory sensitivity characterizes one’s capability to observe weak sensory stimuli. Emotional reactivity is a tendency to respond with intensity to stimuli, which induces emotions. Endurance is an ability to withstand in long-lasting or exhausting conditions. Activity is an inclination to engage in behaviors taking place in intensely stimulating conditions. Briskness is an ability for quick reacting and shifting from one behavior to another. Perseverance is a tendency to repeat emotional states in reaction to stimuli even if the stimulus is no longer present. Functional significance of temperamental characteristics as postulated by the RTT was subject of numerously research projects. FCB-TI has 120 items, 20 items per scale (each scale can yield a total score of 0 to 20). Respondents respond Yes or No to each item. The FCB-TI has good psychometric parameters. Cronbach α vary from 0.72 to 0.86 depending on the scale. In the current study, the range was from 0.71 to 0.82.

Coping styles were assessed with the Polish version (Strelau et al., 2005) of the Coping Inventory for Stressful Situations (CISS) originally constructed by Endler and Parker (1990). The inventory has 48 diagnostic items and measures three types of coping: emotion-oriented, task-oriented, and avoidant. The avoidant style has two dimensions: distraction and social diversion. Cronbach α for the Polish version range from 0.71 to 0.92. In the current study, they ranged from 0.70 to 0.73.

Intensity of PTSD symptoms was measured with PTSD Inventory (PTSD-C) constructed by Strelau et al. (2002). The questionnaire allows for quantitative estimation of PTSD symptoms on two main dimensions: intrusion/hyperarousal (I/H) (recurrent thoughts relating to the traumatic event and causing arousal) and avoidance/numbing (A/N) (avoidance of trauma-related stimuli and weakened response to these stimuli. It has also general scale of PTSD symptoms. The PTSD-C has 30 items. Each item is rated on a 4-point scale from 1 (the symptom is absent) to 4 (the symptom is always present). The inventory has good reliability. Cronbach α for general scale and two subscales is in the range from 0.90 to 0.97. In the current study, they range from 0.70 to 0.80. The instruction provided in the current study refers to the experience of illness as traumatic event.

Quality of life was measured with the use of Polish version of SF-36 questionnaire (Tylka and Piotrowicz, 2009). The inventory contains 36 questions about health and reactions to disease. Two main dimensions of quality of life are measured there. Physical quality of life refers to the physical sphere, from physical activity to pain and its negative consequences for daily activity. Emotional quality of life covers social activity, emotional consequences of restrictions resulting from health condition, level of energy, and tiredness. SF-36 questionnaire provides also general quality of life index. Answers in the inventory are scored on a 0 to 5 points scale. In the polish version, higher scores mean lower quality of life while lower scores mean higher quality of life. The inventory has good reliability with Cronbach α in the range from 0.75 to 0.95. In the current study, they ranged from 0.75 to 0.80.

Table 1 provides descriptive statistics on all interval scales.

**Table 1:** Descriptive statistics for interval scales.

Questionnaires	Variables	*M*	SD	Min	Max
FCB-TI	Briskness	10.92	2.44	7	19
	Perseveration	10.78	2.48	2	18
	Sensory sensitivity	10.16	2.65	4	19
	Emotional reactivity	10.72	3.05	0	24
	Endurance	9.30	2.63	1	17
	Activity	10.45	2.89	1	16
CISS	Task-oriented coping	48.52	6.00	37	73
	Emotion-oriented coping	48.47	6.34	30	64
	Avoidant coping	48.85	5.99	32	64
	Avoidant-distracted coping	24.32	3.64	15	32
	Avoidant-social coping	15.49	2.50	10	23
PTSD-C	Intrusion/arousal	35.98	5.17	17	47
	Avoidance/numbing	36.16	4.63	25	45
SF-36	Physical Qol	57.91	11.27	23	85
	Emotional Qol	30.35	5.87	10	48

*M, mean; SD, standard deviation; min, minimum; max, maximum*.

## Results

In order to conduct statistical analysis, IBM SPSS 24 statistical package was used (SPSS Inc., 2016).

First, descriptive statistics for the demographic characteristic of the sample and for the interval scales were computed. Second, analysis on associations between PTSD, quality of life, and characteristics of the sample was performed.

The main analysis was performed with the use of hierarchical regression analysis. The first block of the model was devoted to control of socio-medical data. Age, sex, living in a small town with number of inhabitants less than 100 thousands, lack of education upper than secondary, being a parent, and duration of the disease longer than 1 year were entered via the stepwise method. Temperamental traits are subject only to slow changes in time. They limit flexibility of dealing with stress in the process of struggling with illness. They also appear first in ontogenetic development, so they were analyzed as primary predictors. Coping strategies were analyzed as secondary predictors. In the second block, the first block of predictors, temperamental traits were analyzed. In the third block, coping styles were entered. Predictors in the second and the third block were also entered with the use of the stepwise method. We analyzed four models, two for PTSD symptoms as explained variables, one for intrusion/arousal symptom cluster and another one for avoidance/numbing, and then two for quality of life, physical and emotional.

### Descriptive Data

Participants were 69 females diagnosed with breast cancer and 60 males diagnosed with lung cancer aged 24–81 years (*M* = 51.77; *SD* = 11.73). Ninety five participants (73.6%) had children. Table 2 presents the frequency distribution for place of residence, educational level, marital status, and duration of illness. The most frequent place of residence was city with number of inhabitants from 1.000 to 100 thousands. The most frequent level of education was secondary. Most participants were married. In most cases, illness lasted from 1 year to 2 years.

**Table 2:** Frequency distribution – place of residence, educational level and marital status, and duration of illness.

Place of Residence	*N*	%
City with number of inhabitants over 100 thousand	48	37.2
City with number of inhabitants from 1.000 to 100 thousand	67	51.9
Small town with number of inhabitants less than 1.000	12	9.3
Missing data	2	1.6

**Level of education**	***N***	**%**

Higher completed	34	26.4
Higher professional	15	11.6
Post-secondary	16	12.4
Secondary	49	38.0
Occupational	14	10.9
Missing data	1	0.8

**Marital status**	***N***	**%**

Married	95	73.6
Informal relationship	15	11.6
Single	19	14.7

**Duration of illness**	***N***	**%**

Less than one year	61	47.3
1–2 years	41	31.8
Longer than 2 years	22	17.1
Missing data	5	3.9

*n, number of participants; %, percentage of the sample*.

### Regression Models

Associations between analyzed variables were analyzed with the use of hierarchical regression analysis. For the sake of nonnormality of univariate distributions bootstrapping was used with 1.000 of bootstrap samples. In order to verify if multicollinearity biased the models variance inflation factors were computed for each predictor. Table 3 presents acquired estimates of regression coefficients in the final models, i.e., after inclusion of the third block along with the 95% confidence intervals.

**Table 3:** Estimates from the regression models explaining levels of PTSD symptoms and quality of life.

Variables	Beta	SE	95% CI	*p*-value	VIF
**Intrusion/arousal**					
Lack of education upper than secondary	-0.18	0.81	-3.48 ÷-0.28	0.023	1.15
Emotion-oriented coping	0.29	0.07	0.09 ÷ 0.36	0.002	1.52
Avoidant-distracted coping	0.27	0.12	0.15 ÷ 0.62	0.003	1.43
**Avoidance/numbing**					
Lack of education upper than secondary	-0.21	0.75	-3.46 ÷-0.46	0.010	1.33
Being a parent	-0.27	0.92	-4.63 ÷-1.02	0.002	1.49
Age	0.17	0.03	0.01 ÷ 0.13	0.043	1.35
Emotion-oriented coping	0.36	0.06	0.17 ÷ 0.37	0.001	1.16
**Physical Qol**					
Duration of the disease longer than one year	0.26	1.95	2.21 ÷ 9.89	0.002	1.05
Sex (men)	0.20	1.91	0.71 ÷ 8.29	0.020	1.05
**Emotional Qol**					
Age	0.29	0.04	0.04 ÷ 0.23	0.001	1.02
Perseveration	0.19	0.20	0.06 ÷ 0.87	0.026	1.09
Emotional reactivity	0.18	0.17	0.04 ÷ 0.70	0.037	1.08

*Beta, standardized regression coefficient; SE, standard error; 95% CI, bootstrap confidence interval; VIF, variance inflation factor*.

The values of VIFs were all below 10, so all four models are acceptable in terms of multicollinearity (Myers, 1990).

Lack of education upper than secondary was negatively related to PTSD symptoms, both intrusion/arousal and avoidance/numbing. Avoidance/numbing was also negatively related to being a parent and positively related to participants’ age.

None of the temperamental traits were statistically significant predictors of PTSD symptoms, so the acquired results did not confirm the hypothesis H1.

Avoidant-distracted coping and emotion-oriented coping were positively related to intrusion/arousal. Emotion-oriented coping was also positively related to avoidance/numbing, which confirmed the hypothesis H2. Emotion-oriented coping and avoidant-distracted coping both explained 20.7% of intrusion/arousal variance. Emotion-oriented coping explained 11.2% of avoidance/numbing variance.

Duration of the disease longer than 1 year and male sex led to lower physical quality of life. Temperamental traits nor coping styles were statistically significant predictors of physical quality of life.

Participants’ age led to lower emotional quality of life. Higher perseveration and higher emotional reactivity led to poorer emotional quality of life. Both explained 8.9% of emotional quality of life variance. The acquired results were in line with the hypothesis H3. However, they did not confirm the hypothesis H4, because the coping styles were not significantly related to quality of life, emotional, nor physical.

## Discussion

The analysis did not reveal any associations between temperamental traits and PTSD symptoms, so the hypothesis H1 was not confirmed, however, the coping styles were related to level of PTSD symptoms, which confirmed the hypothesis H2.

Considering specific situation of patients diagnosed with malignant neoplasms, it seems that the level of PTSD symptoms in this group may depend on their current situation and their perception of the course of the illness. Particular stressful events that are consequences of the disease such as aches after the operation, returning home after hospital stay, disturbances in close social relationships may affect current specificity of coping strategies (Wasteson et al., 2002), but not the temperamental traits, which are not the subject to temporary change. Other situational determinants of coping strategies levels worth considering are the duration of the disease, the incidence of complications during treatment, subjective evaluation of how to improve the health status and satisfaction with treatment or length of hospital stay (Bucholc et al., 2016). The number of possible factors and their importance for patients suffering from possible life-threatening disease leads to conclusion that role of temperamental traits and coping strategies for intensity of PTSD symptoms may be eventually verified only in studies designed to control most of the factors.

Emotion-oriented coping and avoidant distracted coping were found to be associated with higher level of PTSD symptoms. These two strategies were also pointed out as dysfunctional in other research results (Pérez et al., 2014; Richardson et al., 2016), however, the role of emotion-oriented coping was also found to be positive in terms of reducing PTSD symptoms over time (Johnsen et al., 2002). Studies systematically provide data on the positive relationship of emotional coping with stress and symptoms of PTSD. Among styles and strategies to deal with stress, those based on emotions are indicated as unambiguously non-adaptive. Concentration on emotion is associated with increased state of anxiety absorption, increased sense of tension, and anxiety. These emotions are characteristic of traumatic abnormalities – irrespective of the traumatic nature of the trauma – incidental or chronic, a stressor placed outside the person, such as a flood or in the middle, like in case of severe illness. Additional negative emotions are provided by and avoidance strategy. It is possible that avoidance during prolonged stress instead of reducing its level increases intrusive thoughts. Emotion-oriented coping precludes acceptance of the difficult situation of oncological patients. Active coping response is difficult and therefore psychological distress leads to psychopathological symptoms. Emotion-oriented coping is associated with higher state of anxiety and increased tension and both are characteristic for traumatic disorders.

The stress of cancer is a complex phenomenon. Sumalla et al. (2009) in the study of people after oncological treatment draws attention to the multiplicity of stressful stimuli in this disease and difficulties in grasping the most traumatic factor. A similar hypothesis is put forward by Kangas et al. (2002), claiming that diagnosis and treatment of cancer is not a simple trauma in which a reliable causal relationship between different types of stressors and the symptoms of post-traumatic stress disorder can be established. Perhaps in the presented study, trauma symptoms were also associated with other variables, not controlled in the study, especially with those concerning the course of illness and the course of treatment.

The analysis showed that associations between temperamental traits, coping styles and quality of life in the sample of patients diagnosed with cancer were weaker than it was expected. Only emotional reactivity and perseveration were found to be negatively related to emotional quality of life, which was in accordance with the hypothesis H3. Other temperamental traits were not related to quality of life nor to the level of PTSD. The coping styles were related to level of PTSD symptoms but were not related to quality of life, physical, nor emotional, so the acquired results did not confirm the hypothesis H4.

Emotional reactivity and perseveration were found to be factors that were associated with lower emotional quality of life. Highly reactive individuals are characterized by high levels of absorption of negative emotions and anxiety like in neuroticism (Strelau, 2002). Theoretically neuroticism can be connected with high-emotional reactivity and perseveration. The association has also been proved empirically (Zawadzki and Strelau, 2010). The results from the current is therefore consistent with results from other investigators concerned with the role of neuroticism (Härtl et al., 2010; Aarstad et al., 2011; Beisland et al., 2013; Huang et al., 2017). According to RTT people with higher emotional reactivity have reduced capacity threshold and prolonged stressful situations such as chronic disease, potentially life-threatening are especially difficult to bear for them. Perseveration as a tendency to repeat emotional states in reaction to stimuli even if the stimulus is no longer present strengthens the effect of emotional reactivity.

Coping strategies as mentioned above change over time and their significance for quality of life can be difficult to establish with the use of inventories measuring coping as a consistent long-lasting trait. In order to interpret this result once again, one has to be aware of importance of the patients’ perception of their current health condition even when they are in the group of survivors (Watson et al., 2016; Jang et al., 2017). It is possible that when the treatment is perceived as effective and side-effects are minimal quality of life may be satisfactory despite the ineffective stress coping and PTSD symptoms. This matter also needs further research design for controlling more health and treatment status related factors.

The findings of the current study are very different from results obtained in the sample of patients after myocardial infarction (Burnos, 2018, unpublished). The results from that sample showed a complex model showing various relations between various psychological variables. The quality of life depended on many factors. Specifically, higher sensory sensitivity led to lower emotion-oriented coping which in turn lowered PTSD symptoms and improved physical and emotional quality of life. Higher level of briskness also lowered emotion-oriented coping and promoted avoidant-social coping, which also lowered PTSD symptoms and in turn improved quality of life. The results from the current study did not confirm the role of temperamental traits for PTSD symptoms and did not confirm the role of coping styles for quality of life in the studied group. Since both research projects were carried out with the use of exactly the same assessment inventories the differences between them should interpreted in terms of different psychological processes that occur among patients after myocardial infarction and among patients diagnosed with malignant neoplasms.

The situation of patients diagnosed with cancer is specific, because they deal with long-term threat of life. Even if the episode of the disease occurred a long time ago, patients are under pressure of recurrence (Oniszczenko and Laskowska, 2014). It is a prolonged crisis, and it is possible that it induces specific psychological processes. The situation is different from the plight of patients after myocardial infarction where fear of another attack is present initially, but its level decreases over time (Skrzyński, 2006). Patients diagnosed with cancer deal with fear even if the treatment was successful and they are considered cancer survivors (Koch-Gallenkamp et al., 2016).

Clearly the results of the current study do not support the model of psychological processes in which subsequent stages are as follows: temperament – coping styles – PTSD – quality of life although it was supported by the results obtained in the group of patients after myocardial infarction (Burnos, 2018, unpublished). Coping strategies are important factor for PTSD symptoms level in both samples, but in contrary to the patients after myocardial infarction, in the sample of cancer diagnosed patients the role of temperamental traits was minimal.

The presented study has some limitations. The main limitation is lack of control of the specific factors concerned with current health and treatment status. Only duration of illness was measured, and it was done in wide intervals for descriptive purposes. Another limitation is lack of longitudinal data. The data collected during the process of adaptation or progress of the disease could strengthen conclusions. It can also be argued that control of variables concerning health condition in many aspects besides cancer disease, the quality of medical care, and its consequences is needed as well as control of environmental variables including relations with relationships with relatives and loved ones providing support (Luszczynska et al., 2013; Leung et al., 2016). Another important factor decisive for quality of life of patients diagnosed with cancer that was not included in the current study is spirituality. Its role is also underlined in research reports (Laubmeier et al., 2004; Park and Cho, 2017). It was found to reduce symptoms of distress in cancer patients regardless of life threat and to have associations with the level of adjustment.

The current study proofed the role of emotional reactivity and perseveration for emotional quality of life and the role of stress coping for the intensity of PTSD symptoms. Higher level of emotional reactivity, perseveration and higher level of avoidant and emotion-oriented coping were associated with lower level of functioning in the group of patients with cancer.

## Author Contributions

AB and KB-M wrote the Introduction, conceptualized the research, and interpreted the results in the Discussion section. AB carried out the study and analyzed the results.

## Conflict of Interest Statement

The authors declare that the research was conducted in the absence of any commercial or financial relationships that could be construed as a potential conflict of interest. The reviewer MR declared a shared affiliation, with no collaboration, with the authors to the handling Editor at the time of the review.
